# Application Effect of Different Concentrations of Platelet-Rich Plasma Combined with Quadriceps Training on Cartilage Repair of Knee Osteoarthritis

This article has been retracted.

**DOI:** 10.1155/2022/7878064

**Published:** 2022-01-10

**Authors:** Zutong Wu, Jianwen Yin, Yajia Yue, Yiqun Zhang

**Affiliations:** ^1^Department of Orthopedics, The First Affiliated Hospital of Shaoyang University, Shaoyang, 422000, Hunan, China; ^2^Department of Radiology, The First Affiliated Hospital of Shaoyang University, Shaoyang, 422000, Hunan, China

## Abstract

We investigated the application effect of different concentrations of platelet-rich plasma (PRP) combined with quadriceps training on cartilage repair of knee osteoarthritis. Data of 37 patients with knee osteoarthritis (KOA) treated in our hospital (November 2019–February 2021) were retrospectively analyzed and the patients were divided into low concentration group (LCG) (*n* = 12), medium concentration group (MCG) (*n* = 12), and high concentration group (HCG) (*n* = 13) according to the order of admission. All patients received quadriceps training. Three groups above received knee injection of PRP, and the platelet concentrations were 1000–1400 × 10^9^/L, 1400–1800 × 10^9^/L, and 1800–2100 × 10^9^/L, respectively. Articular cartilage thickness of the medial and lateral femur, knee joint function scores, inflammatory factor levels, and matrix metalloproteinases (MMPs) levels were compared. After treatment, compared with the MCG and HCG, articular cartilage thickness of the medial and lateral femur of the diseased side in the LCG was obviously lower (*P* < 0.05). At 2 months after treatment (*T*_3_), compared with the HCG, articular cartilage thickness of the medial and lateral femur of the diseased side in the MCG was obviously higher (*P* < 0.05), without remarkable difference in articular cartilage thickness of the medial and lateral femur of the healthy side among three groups (*P* > 0.05). After treatment, compared with the LCG, knee joint function scores of the MCG and HCG were obviously better (*P* < 0.001). Compared with the HCG, the knee function score at *T*_3_ in the MCG was obviously better (*P* < 0.001). After treatment, compared with the LCG, inflammatory factor levels and levels of MMPs in the MCG and HCG were obviously lower (*P* < 0.05). Compared with the HCG, inflammatory factor levels and levels of MMPs at *T*_3_ in the MCG were obviously lower (*P* < 0.05). PRP combined with quadriceps training can accelerate cartilage repair of patients with KOA and reduce inflammatory factor levels and levels of MMPs, but the treatment effect of PRP depends on platelet concentration, with the best range of 1400–1800 × 10^9^/L. Too high or too low platelet concentrations will affect recovery of knee function.

## 1. Introduction

Knee osteoarthritis (KOA) is an orthopedic disease with knee cartilage degeneration as the main pathological change, which is abnormal metabolism of cartilage matrix together with sterile inflammation of periarticular tissues [1, 2]. With clinical manifestations of knee swelling, pain, and stiffness and decreased knee function, the disease may lead to disability in severe cases, which poses a threat to patients' lives and health. Modern medicine takes repairing articular cartilage as the main idea in the treatment of KOA [3, 4], and oral administration of nonsteroidal anti-inflammatory drugs (NSAIDs) and intra-articular injection of hyaluronan are commonly used in clinic to relieve symptoms [5, 6]. However, in practice, it shows that conventional treatment cannot restore the blood supply of knee cartilage and has a limited effect on promoting articular cartilage repair [7, 8]. With the development of regenerative medicine in recent years, tissue-engineered cartilage has become a new hotspot in the field of cartilage repair in KOA [9]. Most studies believe that PRP can release active substances such as chemokines and growth factors to induce the differentiation from stromal stem cells to chondrocytes in order to promote the synthesis of type II collagen in articular cartilage. At the same time, PRP can also inhibit the breakdown of cartilage by MMPs and reduce the concentration of inflammatory mediators, which has high application value in clinic [10, 11]. However, no unified standard for the use of PRP is found in clinical practice, and a few studies have shown that the efficacy of PRP is not significantly better than the conventional treatment [12]. Some scholars have previously found that PRP is dose-dependent [13]. Whether the limited treatment effect of PRP shown in a few studies is related to its concentration needs to be further explored and confirmed. Redondo M L et al. found that PRP could induce the proliferation of stromal stem cells to chondrocytes, with a positive correlation between PRP concentration and the proliferation rate of chondrocytes [14], which was consistent with the results obtained at *T*_2_ of this study.

In addition, quadriceps training can enhance the stability of the knee joint and mitigate muscle atrophy. By a physical method of squeezing the knee joint, the treatment method can also enhance synovia circulation, improve blood flow of the knee cartilage, and increase the nutrition supply, which facilitates the maintenance of the thickness and strength of the cartilage after drug treatment and enhances knee joint function. The application of PRP combined with quadriceps training may reinforce the application effect of PRP, which changes the view that the curative effect of PRP is not satisfactory in a few previous studies. In this paper, the optimal concentration of PRP is studied based on quadriceps training.

## 2. Materials and Methods

### 2.1. General Information

Data of 37 patients with KOA treated in our hospital (November 2019–February 2021) were retrospectively analyzed. Inclusion criteria were as follows. (1) Patients and their families fully understood the research process and signed the consent form. (2) Patients were diagnosed with degenerative disease of the unilateral knee joint by imaging examination in accordance with the diagnostic criteria of *Guidelines for the Diagnosis and Treatment of Osteoarthritis (2007)* [15]. (3) Patient had knee pain and swelling for more than 6 months and joint fricative in exercise. (4) Patients' Kellgren–Lawrence grade (K-L grade) was between grades I and III [16]. Exclusion criteria were as follows. (1) Patients had mental problems or could not be communicated with. (2) Patients suffered from rheumatoid arthritis in the knee, knee tumors, and *tuberculosis* and intra-articular fractures and were complicated with gout, hematologic diseases, severe cardiovascular diseases, coagulopathy, and liver and kidney dysfunction. (3) Patients had knee joint trauma. (4) Patients' Kellgren–Lawrence grade (K-L grade) was grade 0. (5) Patients used anti-inflammatory analgesics and hormone drugs in recent 1 month [17]. (6) Patients were with acute pain of KOA. (7) Patients were pregnant or lactating. (8) Patients withdrew from the experiment halfway.

A total of 37 patients were included in this study and divided into low concentration group (LCG) (*n* = 12), medium concentration group (MCG) (*n* = 12), and high concentration group (HCG) (*n* = 13) according to the order of admission, with no statistical difference in patients' general data among three groups (*P* > 0.05); see Table 1. The study was approved by the Hospital Ethics Committee.

### 2.2. Withdrawal Criteria

For patients who were in the following situations and were inappropriate to continue the experiment according to the judgment of the research group, their medical record sheets were kept, but the data were not analyzed. (1) Patients experienced adverse events or serious adverse events. (2) Patients presented with deterioration during the experiment. (3) Patients had severe comorbidities or complications. (4) Patients were not willing to continue the clinical trial and asked the research group for withdrawal.

### 2.3. Methods

#### 2.3.1. Quadriceps Training

All patients received quadriceps training. Patients were asked to take a supine position, straighten and raise both legs together, and keep the heel 0.3 m away from the bed for 0.5 min, with a break of 5 s. The actions above were regarded as 1 time and 10 times as a set. 15 sets were required daily, except on the day of injection and the following day, for a total of 2 months.

#### 2.3.2. PRP Treatment

*(1) Fabrication*. 40 ml/(person) time of cubital venous whole blood was collected with a vacuum sterile test tube under strict sterile conditions and anticoagulated with 5 ml of sodium citrate (Taishan Xinning Pharmaceutical Co., Ltd., NMPA approval no. H44024783). The concentrated platelets were separated by PRP method and put into the medical high-speed centrifuge (Yancheng Anxin Experimental Instrument Co., Ltd., specification: AXTD530). PRP was obtained by two-round centrifugation using the Landesberg method. After the first-round centrifugation, the whole supernatant was pipetted into a pipette to 3 mm below the liquid-solid interface. The supernatant was centrifuged again. The second-round centrifugation was performed for 10 min. About 3/4 of the supernatant was removed and discarded, and the rest was shaken to obtain even PRP. (2) Activation: 0.2 ml of PRP was diluted with 0.9% sodium chloride injection (Guangzhou Pearl River Pharmaceutical Co., Ltd., NMPA approval no. H44025125) to 2 ml for later examination. The obtained PRP was diluted with 0.9% sodium chloride to 1000–1400 × 10^9^/L, 1400–1800 × 10^9^/L, and 1800–2100 × 10^9^/L according to the concentration of each group. Then 10% calcium chloride (Sinopharm Group Rongsheng Pharmaceutical Co., Ltd., NMPA approval no. H20065400) was added into 2 ml of PRP in each group to activate platelet in PRP. (3) Treatment: patients were treated with knee injection every week for 2 months, without local anesthesia before injection. After injection, the patients were flexed and extended to exercise the knee joint and then rested in bed for 2 days to avoid excessive walking and strenuous activity.

### 2.4. Observation Criteria

1. Articular cartilage thickness of the medial and lateral femur: the probe frequency of a color Doppler ultrasound instrument (GE Healthcare Voluson P6, NMPA Certified No. 20152062178) was set at 9–12 MHz. Patients were asked to take supine position to expose the knee joint and flex knee at a maximum angle. The cartilage thickness was measured at the front of the medial and lateral femoral condyles. The probe was placed horizontally in the knee joint space to scan the lateral surface of the medial and lateral femoral condyles, and the cartilage thickness of the medial and lateral condyles of the patient was measured on the healthy side and the diseased side before treatment (T1), one month after treatment (*T*_2_), and two months after treatment (*T*_3_).
2. Knee joint function scores: patients' knee joint function at *T*_1_, *T*_2_, and *T*_3_ was evaluated by Lequesne index and Lysholm knee score. The reliability and sensitivity were verified by international literature, and the specific introduction was as follows. (a) Lequesne index [18]: the scale contained 6 items on knee rest pain, pain on movement, tenderness, swelling, and ability to walk, with 0–3 points for the first 5 items, 0–8 points for the sixth item, and a total score of 23 points. Higher scores indicated poorer knee function. (b) The Lysholm knee score [19] formulated by Lysholm and Gillqui: the scale was an 8-item questionnaire measuring pain, instability, locking, swelling, limp, stair-climbing, squatting, and use of support, with a total score of 100 points. Below 65 points represented poor knee joint function, 65–84 points represented medium knee joint function, 85–94 points represented good knee joint function, and above 95 points represented excellent knee joint function.
3. Inflammatory factor levels: at *T*_1_, *T*_2_, and *T*_3_, patients were asked to take supine position, and 5 ml of fasting venous blood was collected from the patients in the morning with routine local disinfection and local anesthesia (Lidocaine, Fujian Kinsan Bio Pharmaceutical Co., Ltd., NMPA approval no. H35020528). 2 ml of synovial fluid was withdrawn from the joint cavity by puncturing the syringe just above the patella and lateral quadriceps femoris. Interleukin-1 *ß* (IL-1*β*), interleukin-6 (IL-6), and tumor necrosis factor *a* level (TNF-*α*) were measured by enzyme-linked immunosorbent assay (ELISA) (Beijing Kewei Clinical Diagnostic Reagent Co., Ltd., NMPA approval no. S20060028). Erythrocyte sedimentation rate (ESR) was measured by Westergren method (Shanghai Yaji Biotechnology Co., Ltd., NMPA certified no. 20163400149).
4. Levels of MMPs: at *T*_1_, *T*_2_, and *T*_3_, synovial fluid above was collected for detection of matrix metalloproteinase-1 (MMP-1), matrix metalloproteinase-3 (MMP-3), matrix metalloproteinase-9 (MMP-9), and matrix metalloproteinase-13 (MMP-13) by ELISA.

### 2.5. Statistical Processing

In this study, the data were processed by SPSS20.0 and graphed by GraphPad Prism 7 (GraphPad Software, San Diego, USA). Including enumeration data and measurement data, the study used X2 test and *t*-test. The differences were statistically significant at *P* < 0.05.

## 3. Results

### 3.1. Comparison of Articular Cartilage Thickness of the Medial and Lateral Femur

After treatment, compared with the MCG and HCG, the articular cartilage thickness of the medial and lateral femur of the diseased side in the LCG was obviously lower (*P* < 0.05). Compared with the HCG, articular cartilage thickness of the medial and lateral femur of the diseased side in the MCG at *T*_3_ was obviously higher (*P* < 0.05), without remarkable difference in articular cartilage thickness of the medial and lateral femur of the healthy side among three groups (*P* > 0.05); see Figure 1.

Figure 1(a) shows the articular cartilage thickness of the medial and lateral femur, with no obvious difference in the articular cartilage thickness of the medial and lateral femur of the diseased side in the LCG, MCG, and HCG at *T*_1_ (2.77 ± 0.11 vs. 2.74 ± 0.10 vs. 2.71 ± 0.12, *P* > 0.05). Compared with the MCG and HCG, the articular cartilage thickness of the medial and lateral femur of the diseased side in the LCG at *T*_2_ and *T*_3_ was remarkably lower (2.84 ± 0.10 vs. 2.96 ± 0.12 vs. 3.04 ± 0.12, 2.90 ± 0.10 vs. 3.34 ± 0.13 vs. 3.10 ± 0.12, *P* < 0.05). Compared with the HCG, the articular cartilage thickness of the medial and lateral femur of the diseased side in the MCG at *T*_3_ was remarkably higher (3.34 ± 0.36 vs. 3.10 ± 0.32, *P* < 0.05).

Figure 1(b) shows the articular cartilage thickness of the medial and lateral femur of the healthy side, with no obvious difference in the articular cartilage thickness of the medial and lateral femur of the healthy side in the LCG, MCG, and HCG at *T*_1_, *T*_2_, and *T*_3_ (3.30 ± 0.12 vs. 3.32 ± 0.10 vs. 3.31 ± 0.11, 3.25 ± 0.10 vs. 3.28 ± 0.11 vs. 3.27 ± 0.12, 3.26 ± 0.11 vs. 3.29 ± 0.13 vs. 3.28 ± 0.10, *P* > 0.05).

### 3.2. Comparison of Knee Joint Function Scores

Compared with the LCG, Lequesne indexes and Lysholm knee scores in the MCG and HCG were remarkably better (*P* < 0.001). Compared with the HCG, Lequesne indexes and Lysholm knee scores of MCG at *T*_3_ were remarkably better (*P* < 0.001); see Figure 2. Compared with the LCG, the MCG and HCG achieved more ideal effect in cartilage repair, and the inflammatory factor levels and levels of MMPs in the two groups were conspicuously lower (*P* < 0.05), demonstrating that PRP can inhibit the action of MMPs, reduce the degradation ability of extracellular matrix, and balance the gene expression of inflammatory mediators, but the therapeutic effect knits a close connection to the platelet concentration.

Figure 2(a) shows Lequesne indexes, with no significant difference in Lequesne indexes at *T*_1_ in LCG, MCG, and HCG (9.54 ± 0.63 vs. 9.56 ± 0.64 vs. 9.60 ± 0.61, *P* > 0.05). Compared with the MCG and HCG, Lequesne indexes in LCG at *T*_2_ and *T*_3_ were remarkably higher (6.54 ± 0.41 vs. 5.23 ± 0.31 vs. 5.10 ± 0.35, 5.10 ± 0.21 vs. 4.02 ± 0.20 vs. 4.56 ± 0.24, *P* < 0.001). Compared with the HCG, Lequesne indexes of MCG at *T*_3_ were remarkably lower (4.02 ± 0.20 vs. 4.56 ± 0.34, *P* < 0.001).

Figure 2(b) shows Lysholm knee scores, with no obvious difference in Lysholm knee scores at *T*_1_ in LCG, MCG, and HCG (54.85 ± 2.35 vs. 54.68 ± 2.51 vs. 54.75 ± 2.31, *P* > 0.05). Compared with the MCG and HCG, Lysholm knee scores in LCG at *T*_2_ and *T*_3_ were remarkably lower (60.10 ± 2.15 vs. 78.98 ± 2.54 vs. 80.22 ± 2.41, 70.54 ± 2.68 vs. 90.23 ± 2.65 vs. 84.21 ± 2.41, *P* < 0.001). Compared with the HCG, Lysholm knee scores in MCG at *T*_3_ were remarkably higher (90.23 ± 2.65 vs. 84.21 ± 2.41, *P* < 0.001).

### 3.3. Comparison of Inflammatory Factor Levels

After treatment, compared with the LCG, inflammatory factor levels in MCG and HCG were remarkably lower (*P* < 0.05). Compared with the HCG, inflammatory factor levels in the MCG were remarkably lower (*P* < 0.05); see Table 2.

### 3.4. Comparison of Levels of MMPs

After treatment, compared with the LCG, levels of MMPs in MCG and HCG were remarkably lower (*P* < 0.05). Compared with the HCG, levels of MMPs in MCG at *T*_3_ were remarkably lower (*P* < 0.05); see Table 3.

## 4. Discussion

The main pathological changes of KOA are the progressive changes of articular cartilage. Patients have reduced cartilage extracellular matrix and reduced knee cartilage function and lack a stable blood supply, which is difficult to complete self-repair after damage, so inhibiting the reduced cartilage extracellular matrix and improving the blood supply at the cartilage are crucial to repair articular cartilage. KOA involves articular cartilage, synovium, ligaments around the joint and muscle groups, so patients often have quadriceps atrophy, which results in the imbalance of the tension between the medial and lateral of the patella, biomechanical disorder of the patella joint, and disuse atrophy of the muscles and aggravates KOA to some extent. Therefore, quadriceps training has always been the emphasis of the KOA treatment. The latest research shows that the training can break the vicious cycle of joint instability, promote the local venous and lymphatic reflux near the joint, improve the clearance of pain-causing factors in the joint cavity, restore the nutrition supply of articular cartilage, maintain cartilage thickness restored by drug treatment [20], and then accelerate the process of knee functional rehabilitation. In this study, quadriceps training was used as the basic treatment method. It was found that the cartilage thickness of the three groups after treatment was conspicuously better than that before treatment, and the cartilage thickness of the LCG after treatment was (2.84 ± 0.10) mm, which was also obviously higher than that of the experimental group using PRP at the concentration of 1500–1800 × 10^9^/L in the study of scholar Naveed et al. [21]. It indicated that quadriceps training could enhance the cartilage repair effect of PRP and stabilize the treatment effect.

However, with longer treatment time, the cartilage repair rate of the diseased side in MCG gradually exceeded that in the HCG, which demonstrated that the treatment effect of the drug gradually decreased when the concentration of platelet in the PRP was above the optimal value. The reason may lie in the fact that some of the cytokines in PRP have a negative effect on KOA treatment. For example, transforming growth factor *ß* (TGF-*β*) is beneficial for cartilage repair, but an excessive amount will weaken the synthesis of bone morphogenetic protein (BMP) and reduce the differentiation rate of chondrocytes [22]. In addition, compared with the HCG, inflammatory factor levels and MMPs in the MCG at *T*_3_ were conspicuously lower (*P* < 0.05), which may be related to release of more leucocytes by platelets at the high concentration. Inflammatory mediators such as interleukin and MMPs can affect the synovial joints of patients and aggravate the sense of joint pain [23]. Therefore, the knee function scores in the HCG were lower at *T*_3_, showing that PRP at the concentration of 1800–2100 × 10^9^/L impacts on patients' long-term quality of life, which is not conducive to the recovery of knee function.

## 5. Conclusion

It is worth noting that this study only analyzed the data of patients at 2 months after treatment. After analysis of the laboratory data of patients with KOA at 6 months after the application of PRP, some scholars found that when the platelet concentration was 1500–1800 × 10^9^/L, the curative effect was more obvious at 2–3 months after treatment. However, the knee function maintenance effect of patients in HCG was better at 6 months after treatment. It is speculated that the content of active substances was more in high concentration of PRP, but lower in low and medium concentration, which was completely released at 6 months, and the effect was no longer obvious [24]. Although some differences are found in the experimental results of different studies, it is suggested that there is the best application concentration of PRP [25]. From the results of this study, 1400–1800 × 10^9^/L is the best application concentration, which can significantly benefit patients in the short term, but the long-term efficacy still needs further exploration.

To sum up, PRP combined with quadriceps training can accelerate cartilage repair of patients with KOA and reduce inflammatory factor levels and levels of MMPs, but the treatment effect of PRP depends on platelet concentration, with the best range of 1400–1800 × 10^9^/L. Too high or too low platelet concentrations will affect recovery of knee function.

## Figures and Tables

**Figure 1:** Comparison of articular cartilage thickness of the medial and lateral femur ( $\bar{x}\pm s$, mm). *Note.* The abscissa from left to right was *T*_1_, *T*_2_, and *T*_3_, respectively, and the ordinate was thickness (mm). The black area was LCG, the dark gray area was MCG, and light gray was HCG. # indicated *P* < 0.05.

**Figure 2:** Comparison of knee joint function scores ( $\bar{x}\pm s$, points). *Note.* The abscissa from left to right was T_1_, T_2_, and T_3_, respectively. The black area was LCG, the dark gray area was MCG, and light gray was HCG. # indicated *P* < 0.001.

**Table 1:** Comparison of general data of patients.

Group	LCG (n = 12	MCG (n = 12	HCG (n = 13	P
*Gender*				
Male	7	7	8	>0.05
Female	5	5	6	
*Age (years)*				
Range	41–74	41–72	40–75	
Average age	62.65 ± 1.23	62.45 ± 1.20	62.56 ± 1.25	>0.05
Average course of disease	5.87 ± 1.10	5.89 ± 1.23	5.85 ± 1.20	>0.05
*Diseased sides*				
Left	7	8	8	>0.05
Right	5	4	5	
Mean body mass (kg)	56.12 ± 2.15	56.23 ± 2.10	56.18 ± 2.05	>0.05
BMI (kg/m^2^)	21.98 ± 2.10	21.89 ± 2.15	21.95 ± 2.13	>0.05
*K-L grades*				
I	6	6	7	>0.05
II	3	4	3	
III	3	2	3	
IKDC score^*∗*^	53.65 ± 5.14	53.60 ± 5.10	53.34 ± 5.15	>0.05
WOMAC score^*∗∗*^	28.95 ± 5.10	28.92 ± 5.23	28.89 ± 5.10	>0.05
*Education degree*				
Middle school degree and below	2	3	4	>0.05
Senior high school or junior college degree	6	6	7	
University degree and above	4	3	2	
*Monthly income (yuan)*				
≥3000	6	7	7	>0.05
＜3000	6	5	6	
*Marital status*				
Married	9	10	9	>0.05
Unmarried, divorced, or widowed	3	2	4	
*Residence*				
Rural	7	6	8	>0.05
Urban	5	6	5	

*Note.* ^*∗*^ The score of International Knee Documentation Committee (IKDC). ^*∗∗*^Osteoarthritis index score of Ontario University and McMaster University.

**Table 2:** Comparison of inflammatory factor levels ($\bar{x}\pm s$ ).

Group	LCG (*n* = 12)	MCG (*n* = 12)	HCG (*n* = 13)
*T*_*1*_			
IL-1*β* (pg/ml)	80.11 ± 6.34	80.41 ± 6.21	80.23 ± 6.24
IL-6 (ng/ml)	170.54 ± 10.21	171.65 ± 10.41	170.98 ± 10.32
TNF-*α* (pg/ml)	90.23 ± 5.41	90.54 ± 5.23	90.35 ± 5.24
ESR (mm/h)	20.11 ± 2.12	20.65 ± 2.10	20.45 ± 2.13

*T2*			
IL-1*β* (pg/ml)	68.98 ± 3.54	51.98 ± 3.20^#^	50.78 ± 3.23^#^
IL-6 (ng/ml)	130.54 ± 12.68	105.41 ± 10.44^#^	104.98 ± 10.65^#^
TNF-*α* (pg/ml)	60.98 ± 2.15	48.12 ± 2.65^#^	47.95 ± 2.54^#^
ESR (mm/h)	16.55 ± 1.54	11.98 ± 1.41^#^	10.99 ± 1.23^#^

*T3*			
IL-1*β* (pg/ml)	42.98 ± 2.15	30.14 ± 2.33^#^	36.54 ± 2.14^###^
IL-6 (ng/ml)	96.84 ± 2.65	82.12 ± 2.45^#^	88.64 ± 2.14^###^
TNF-*α* (pg/ml)	46.12 ± 2.57	28.32 ± 1.54^#^	32.88 ± 2.54^###^
ESR (mm/h)	9.90 ± 0.51	8.23 ± 0.45^#^	8.70 ± 0.65^###^

*Note.* # indicated *P* < 0.05 compared with LCG, and ## indicated *P* < 0.05 compared with MCG.

**Table 3:** Comparison of levels of MMPs ( $\bar{x}\pm s$ ).

Group	LCG (*n* = 12)	MCG (*n* = 12)	HCG (*n* = 13)
*T*_*1*_			
MMP-1 (*μ*g/ml)	0.60 ± 0.05	0.61 ± 0.05	0.63 ± 0.04
MMP-3 (ng/ml)	230.98 ± 12.15	231.98 ± 12.40	229.98 ± 12.01
MMP-9 (ng/ml)	70.54 ± 2.68	70.68 ± 2.41	71.01 ± 2.35
MMP-13 (ng/ml)	298.65 ± 12.41	297.41 ± 10.57	300.10 ± 13.14

*T2*			
MMP-1 (*μ*g/ml)	0.56 ± 0.04	0.46 ± 0.06^#^	0.44 ± 0.04^#^
MMP-3 (ng/ml)	170.54 ± 8.54	135.20 ± 6.98^#^	130.65 ± 6.55^#^
MMP-9 (ng/ml)	55.24 ± 3.54	43.20 ± 2.15^#^	42.11 ± 2.68^#^
MMP-13 (ng/ml)	240.21 ± 12.68	205.98 ± 10.41^#^	200.68 ± 12.14^#^

*T3*			
MMP-1 (*μ*g/ml)	0.42 ± 0.04	0.31 ± 0.04^#^	0.38 ± 0.05^###^
MMP-3 (ng/ml)	96.84 ± 2.65	82.12 ± 2.45^#^	88.64 ± 2.14^###^
MMP-9 (ng/ml)	38.54 ± 3.22	29.68 ± 2.10^#^	34.12 ± 2.12^###^
MMP-13 (ng/ml)	156.98 ± 12.41	137.68 ± 10.45^#^	146.68 ± 10.41^###^

*Note.* # indicated *P* < 0.05 compared with LCG, and ## indicated *P* < 0.05 compared with MCG.

## Data Availability

The datasets used and/or analyzed during the current study are available from the corresponding author on reasonable request.
